This article has been retracted.

# Cluster Analysis Algorithm in the Analysis of College Students' Mental Health Education

**DOI:** 10.1155/2022/6394707

**Published:** 2022-04-18

**Authors:** Wanting Zheng

**Affiliations:** School of Clinical Medical Technology, Sichuan Vocational College of Health and Rehabilitation, Zigong, 643000 Sichuan, China

## Abstract

With the rapid development of curricula, a large number of studies are emerging to assist in the development of curricula. But in an information society, in the face of rapid learning and increased life expectancy, students face the pressure not to forget; the mental health status as a result of our curricula is closely related to our learning. The research and application of the integration algorithm plays an important role in the analysis of the mental health education system. The purpose of this work is to study the application analysis algorithm in the students' context. This work applies the integration analysis algorithm to students' mental health analysis and identifies students' mental health problems using the integration analysis algorithm so that students are well informed and guided. Based on the system engineering method, using the data mining clustering method, a detailed analysis and research on the mental health of college students is done. In this work, a method of student behavior analysis and statistical tools are used to collect mental health data to find common features of different groups of students, in order to better visualize and investigate the mental health of these students on a scientific basis. The results of this study are as follows: a general analysis algorithm application on the analysis of students' mental health education system allows for an effective understanding of scientific data. FCM and FCM algorithms based on the density of information entropy characteristics were used to investigate the effect of mental health factors on the results of the study and the practicality of the algorithm used, which provided an effective method for the prevention of student mental problems. Assisting the school in formulating corresponding new methods of early prevention and intervention of college students' psychological disorders will create a good and healthy atmosphere for college students' study and life. The research results provide a reliable basis for managing and cultivating students.

## 1. Introduction

Mental health education [1] plays an important role in the general development of students. Strengthening and improving the mental health education of college students is an important measure to fully implement the Party's educational policy and promote quality education under the new form. It is an important way to promote the healthy growth of college students and cultivate high-quality qualified talents. Through the mental health education system, students instill learning [2] in their beliefs and externalize them in their own behaviors. The goals in promoting the general development of college students is so that they will have a noble personality, a good understanding of health and good academic quality [3], and a strong scientific ability to adapt. Although the mental health education system in universities and colleges has grown rapidly and some progress has been made in China, there is still a gap in the way mental health education [4] has developed in countries. There are also weaknesses that need to be addressed. On the one hand, the research content of mental health education in colleges and universities in China is flexible. Assessing and understanding the mental health status of college students [5] cannot prevent and intervene effectively in students' mental disorders [6]. On the other hand, the mental health education of most college students is for individuals, not for all students. There is a lack of comprehensive research on the general rule of mental health problems of college students, and mental health consultations are conducted for individual students with mental disorders [7]. In addition, existing research findings may not fully address the various problems facing the mental health system of college students. In general, the research level of mental health education of college students has not reached a certain level, the research methods are incomplete, and the content of the study is insufficient. Therefore, it is necessary to further develop the mental health education system of college students in China and to conduct scientific in-depth training of the medical system. In terms of boosting the general quality of college students [8], colleges and universities should have a quality mental health education system as their primary concern. Currently, there are also some weaknesses in China's mental health education system, which may not provide comprehensive mental health education services for students [9]. This paper hopes that through research on students' mental health education, it can play a positive role in the growth and development of students' mental health education so that young people can meet problems of different parts of society and make efforts and contributions [10, 11]. The basic idea of cluster analysis is to classify samples according to the principle of “clustering together.” The clustering analysis method is an unsupervised learning process; it aggregates things into classes according to some attributes, so that the similarity between different classes is as small as possible, and the similarity between the same classes is as large as possible, so as to realize the classification of data. Cluster analysis can be used as a separate algorithm or as a preprocessing step in other data mining algorithms. Therefore, it is an important research topic in the field of data mining. Cluster analysis techniques have been widely used in many applications, including pattern recognition, data analysis, image processing, and market research. Through clustering, one can identify dense and sparse regions and thus discover global distribution patterns and interesting interrelationships between data attributes.

In recent years, due to the frequent occurrence of malignancies caused by students' mental disorders, the mental health status of students has become the focus of public attention. Experts at home and abroad have done a lot of in-depth research and are actively researching for a scientific guide with involvement of college students. Some developed countries attach great importance to the psychology of young people. They use techniques, methods and measurement tools, and mathematical calculations to analyze students' scientific data [12], in order to teach science coaching teachers to provide targeted scientific guidance to students. They have had a lot of success that is worth learning. Currently, more and more attention is being paid to the mental health education system of college students in China. The in-depth research on the mental health of college students and the exploration of the psychological intervention mode of college students are the focus of domestic and foreign scholars. Local education departments and colleges and universities have done a lot of work in the development of mental health education for college students and carry out corresponding teaching, education, scientific research, and practical activities. At the same time, education departments of all levels have performed many functions in the student mental health education system, such as the establishment and maintenance of the mental health education system and counseling centers and appropriate operating procedures, provision of mental health counseling, and through a wide range of assessments and assessments [13, 14], emphasizing the importance of management and quality education in the mental health system of students. During the Fifth Annual Program, the main research areas are the mental health training of students and teachers, attention to the scientific characteristics and manifestations of Chinese brain barriers [15], and the promotion of academia and a method of psychological counseling suitable for Chinese. To improve the level of scientific research and provide scientific guidance for practice, the following steps should be taken: establishing a network of mental health professionals, promoting research methods, and sharing resources to improve the overall level of research on mental health in China. Mental health research in colleges and universities should be improved, to enable scientific knowledge in a more open, intellectual, and scientific way; to learn from foreign mental health research methods, in combination with national conditions, cultural background, and intellectual characteristics of students; and to explore the cultural diversity of creation, famous improvements and applications of research results, scientific improvements, innovations, and practicality of research. We should strengthen scientific and practical research of scientific knowledge and explore the school mental health education system with Chinese characteristics.

Since the 1980s, Chinese researchers have studied the mental health problems of students, researched the field on different groups of students, and investigated the impact of family and society on different groups of students with anxiety [16], depression [17], self-deprecating behavior, and other behavioral problems [18] and tested the sedation on a small scale and achieved positive results. However, there are still many weaknesses: there is little application of research results to science and psychotherapy and scientific and practical research on psychotherapy and psychotherapy for college students is also recent. Compared to college students, most college science teachers do not have the science, planning, and professional skills. It is difficult for students to acquire and apply science, and the outcome is not clear. It is a quick and important task to find the best psychology for students to manage, to guide them to analyze themselves [19], to understand each other more accurately, to develop themselves, to promote the health of their character [20, 21], to maintain mental health, and to promote good behavior. Mental health education for international college students begins early. Many universities in Europe, the United States, Japan, and other countries have set up mental health service centers for students [22]. Mental health education began in Hong Kong in the 1970s, in Taiwan in the 1950s, and on the mainland in the 1980s.

This work systematically introduces the application of a comprehensive analysis algorithm to the student mental health system and applies it to the student mental health education system in China. In the process of mental health education, the role of teachers is to help students understand their own situation and to help them find their own healthy way of communicating, so that they can go further in their communication. The research content of the mental health education system in colleges and universities in China is flexible. Training and understanding students' mental health cannot effectively prevent and intervene in students' mental health problems. Most student mental health education programs are for individuals, not all students [23]. At the same time, the results of previous research may not solve the mental health problems students face. In general, the research level of mental health education of students has not reached a certain level, the research methods are not systematic, and the content of the study is incomplete. Therefore, there is an urgent need to further develop the mental health education system of college students in China. In order to ensure the effective implementation of mental health education for students, an in-depth study on the mental health education system should be conducted. Combining science with practice, from science and political discipline, in conjunction with specific methods and content of science fiction, and based on science and politics, this paper analyzes the factors that affect the mental health of students, avoiding simple science [24]. This work is a form of questionnaire research, which is a complete and accurate understanding of current students' scientific problems and promotes a larger approach to health education in colleges and universities. To analyze the specific spatial distribution of the data, a two-step clustering analysis algorithm was used. At the same time, the theoretical rationality of the algorithm is clarified, and the data analysis test is made, which can solve the problem of irregular spatial distribution of data to a certain extent. According to the algorithm model proposed above, a cluster analysis model is constructed, and the algorithm is applied to the mental health counseling of college students. After a long period of algorithm research, framework design, and programming implementation, a complete mental health counseling system has been formed, which provides scientific, objective, and reliable data guaranteed for the correct implementation of decision-making strategies. This kind of cluster analysis is integrated into the mental health analysis of college students, so that the school can better understand and grasp the information of students in all aspects.

## 2. Cluster Analysis and Mental Health Education of College Students

### 2.1. Background Knowledge of Cluster Analysis

Clustering is to group data objects into multiple clusters, so that objects in the same cluster have high similarity (similarity), while objects in different clusters have very large dissimilarity (dissimilarity). A good clustering method should produce clustering results with the following characteristics: objects within clusters are highly similar (high intraclass similarity), while objects between clusters are rarely similar (low interclass similarity).

Clustering is a data processing method with a long history, and its importance and wide application have been affirmed by researchers. Clustering is an important part of machine learning and plays an important role in identifying the internal structure of data. Clustering is widely used in data mining [25, 26], image segmentation, data compression, machine vision, and other fields. In today's society which emphasizes big data and intelligent production, the role of clusters is particularly important. Clustering is a method of grouping or clustering data sets according to some inherent characteristics of data sets or the similarity between data samples. The data processed by clustering is usually unmarked, so clustering is an unsupervised machine learning method. Clustering has been widely used in practical production and research. It can not only be used to explore the internal spatial structure of unlabeled data sets but also play an auxiliary role in the data processing stage of other machine learning tasks. Data mining is the process of extracting hidden, unknown, but potentially useful information and knowledge from a large amount of random, noisy, fuzzy, and incomplete data. There are many terms similar to this term, such as knowledge discovery from databases, data analysis, knowledge extraction, pattern analysis, data archaeology, data collection, information harvesting, business intelligence, data fusion, and decision support.

### 2.2. Clustering Algorithm

The basic problem of clustering is how to measure the similarity between sample data. Most of the common clustering algorithms use a certain distance to define the similarity between samples. The closer the distance, the higher the similarity. Dist (Xi, XJ) is the distance function between samples [27]. Clustering should have a clear mining target. Data mining is not a panacea; it must be determined under certain themes in order to play a better effect. First, classify the students with psychological problems and then mine them; secondly, according to the students' psychological problems, select and identify these data from a large number of data in the school, so as to facilitate the effective processing of the data and make it suitable for mining tools.

In practical research and application, the distance used to measure the similarity does not have to strictly meet the above four basic properties. The order distance proposed in the literature based on similarity ranking does not satisfy symmetry and triangle inequality. The image classification algorithm based on this measurement method has achieved good results. In practical tasks, researchers can analyze the data according to the data samples and the problems to be solved and use the appropriate distance calculation function. The following is the similarity measurement method used in this paper: value difference measurement (VDM)—sample attributes can be divided into ordered attributes and disordered attributes [28]. There is a certain size relationship between sorted attributes, and the distance can be calculated directly according to the attribute value. For example, the definition domain of an attribute is {1,2,3,4,5}, which makes it easy to calculate the distance between “1” and “5.” Ordered attributes can be continuous or discrete. However, unordered attributes are usually discrete, and the distance between samples cannot be calculated directly according to the attribute values. For example, the domain of attribute definition is {Ningxia, Tianjin, Nanjing}, and the similarity between attribute values cannot be directly calculated by Euclidean distance. You need to use VDM to calculate the distance between these unordered attributes. The premise of using VDM is that the data has a category label [29].

Based on different training methods, the most commonly used computational algorithms can be divided into five categories: computational compaction, compact compaction algorithm, weight-based algorithm, lattice-based algorithm, and basic composite algorithm. There are generally three steps in the cluster analysis algorithm: feature extraction, algorithm selection, and parameter setting. The main clustering algorithms can be divided into the following categories: partitioning method, hierarchical method, density-based method, grid-based method, model-based method, and fuzzy clustering algorithm (fuzzy clustering methods).

### 2.3. Meaning of Mental Health

Most experts and scholars describe the standard of mental health not only as a single but also as multiple. This is because the performance of mental health is diverse, so it is impossible to use a simple standard to measure everyone, so the standard should be compound. It is generally believed that people who meet the following conditions are mentally healthy.

1. Be able to correctly evaluate themselves, give full play to their strengths and overcome their shortcomings
2. Aware of their responsibility to the country and society, work hard and study hard
3. Be willing to communicate with others, be strict with yourself and lenient to others
4. Able to observe the environment comprehensively and have strong ability to adapt to the environment
5. Good at controlling their own emotions and have strong psychological endurance to setbacks and conflicts

Currently, more and more attention is being paid to students' academic status and mental health system. However, at present, our focus on this project may not meet the brain-changing needs of college students. Although many colleges and universities have set up counseling centers for college students' mental health programs, they have also conducted mental health consultations in many areas. More and more attention is being paid to the mental health problems of students. The problems of mental health education have been successfully addressed. We can better understand the curriculum for students' mental health, curriculum, and lifestyle and the development of their general quality. However, there is not much research on the mental health problems of college students in China, such as lack of fitness, lack of planning, inadequate resources, and inadequate funds. Although mental health facilities have been set up in China, the current situation is worrying. For example, a consulting center was set up at the Beijing University Hospital. If students want to learn about mental health problems, of course, they will think they are sick before they go there. This practice allows students to go to the center only if they think they are ill. The behavior of the school left students confused about mental illness, which led to more brain barriers.

### 2.4. Personality Questionnaire for College Students

The College Student Questionnaire (UPI) is an important measure for measuring the mental health level of college students [30]. The behavioral questionnaire of college students is used primarily to assess students' mental health status, to assess their mental problems, to create mental records of encounters, and to monitor that the health status of the brain of the students is strong. It can help scientists or counselors identify the subject of the problems quickly so that schools can provide timely psychological counseling services to students with disabilities like depression and develop appropriate mental health measures.

UPI consists of three parts: the first part is the basic information of students. It includes students' name, gender, age, address, contact information, family status, interests and hobbies, and enrollment motivation. The second part is the UPI questionnaire itself. It consists of 60 projects. Among them are 4 projects with title numbers of 10, 20, 30, and 40. The other 56 items reflect the students' distress, anxiety, contradiction, and other symptoms. The third part is additional questions, mainly to understand the overall evaluation of their own physical and mental health, whether they have received psychological counseling, and what kind of consultation requirements.

#### 2.4.1. Evaluation and Classification of UPI Results

1. Class A screening criteria

Those who meet one of the following conditions are classified as class A: (1) the total score is more than 26 points (including 26 points), (2) the affirmative choice is made in question 25, (3) there are at least two affirmative options in the auxiliary questions, and (4) those who explicitly ask for consultation are classified as having psychological problems.

(2) Class B screening criteria

Those who meet the following conditions are classified as class B: (1) the total score is between 20 and 24, (2) one of the 81625 questions is a positive choice, and (3) only one auxiliary question is a positive choice.

(3) Class C screening criteria

People who do not belong to the first or second category are classified as class C.

The following characteristics can be used for diagnosis: class A—all kinds of neurosis (phobia, obsessive-compulsive disorder, anxiety disorder, severe neurasthenia, etc.), schizophrenic tendency, pessimism, and strong psychological conflict, obviously affecting normal life and learning. Make an appointment for the next consultation immediately and interview once a week or every other week until the symptoms are relieved. Class B: there are general psychological problems, such as uncoordinated interpersonal relationship and maladjustment to the new environment. These students have all kinds of troubles, but they can still maintain normal study and life. Help them and ask them if they have any questions. The rest are class C, which can prevent them from being interviewed. Their symptoms are temporarily not obvious or have been resolved. If they develop symptoms in the future, they know that counseling can help.

### 2.5. Cattell's 16 Personality Factor Test

Cattel's 16 personality factor test (16PF) has an important influence in the world [31]. They were compiled by the most famous psychologist in the United States, Cattell. Sixteen personality factor tests included gregariousness (a), intelligence (b), stability (c), bullying (e), excitability (f), persistence (g), boldness (h), sensitivity (i), skepticism (l), fantasy (m), and complexity (n). The test has 186 questions and is widely used in the field of career guidance and personnel selection. 16 personality factors are independent.

## 3. Cluster Analysis Algorithm Design

Cluster analysis steps: although the diversity of clustering analysis criteria leads to different clustering results, almost all clustering methods must follow the following steps:

1. *Data preparation*: data preprocessing
2. *Feature selection and extraction*: select effective features to keep as much information as possible in the processed data
3. *Clustering*: select the appropriate clustering algorithm according to the data structure and characteristics
4. *Clustering effectiveness evaluation*: select the appropriate cluster effectiveness index to verify the clustering results
5. *Results analysis*: combined with different experimental data, the clustering results were analyzed and the correct conclusion was obtained

In the above four steps, the selection of the clustering algorithm and clustering effectiveness index will directly affect the validity and correctness of clustering results [32].

The classification standard of cluster analysis is determined by the similarity of data. In order to measure the difference between data elements more accurately, it is necessary to determine the similarity measurement of data elements. The main similarity measures include distance measure, similarity measure, and match measure. Among them, distance measurement is the most common. Since most data elements are multidimensional and vector elements, data elements are called vectors. Their attributes are components, while data sets are vector sets. The distance measure is based on the distance between two vectors. The smaller the distance difference, the higher the similarity between the two vectors. Suppose that vector *x* is an *n*-dimensional data element, that is, *x* = {*X*_1_, *X*_2_, *X*_*n*_}, and *y* is the equivalent *n*-dimensional vector, *y* = {*Y*_1_, *Y*_2_, *Y*_*n*_}, then *d*(*x*, *y*) is defined as the distance between two vectors.

## 4. Application of Cluster Analysis Algorithm in the Analysis of College Students' Mental Health Education

### 4.1. Data Sources

A total of 2012 students from the departments of foreign languages, Chinese, computer science, chemical engineering, economic management, social science, civil engineering, and art took part in the psychological test. The main reference is the effective test data in 2010.

### 4.2. Data Preprocessing

1. These characteristics do not affect the listing results but increase the computational complexity and we eliminate these characteristics directly in the compilation process
2. *Data deletion*: data deletion refers to the lost values of certain data assets. For example, for a small amount of data, according to the data charge law, add a value to the lost value. For large volumes of data, the lost value can be replaced by frequency
3. *Data conversion*: the attribute code conversion table of psychological test data required in this paper is as follows

Table 1 is the attribute code table of a student, and the attribute codes of gender, family income, single parent family, only child, achievement, and personality characteristics are selected.

For the establishment of college students' psychological database and data table, in the process of cluster analysis, the first step is to collect data, and then through data preprocessing, clear up the invalid data, establish the mental health database of college students, and establish the data table. The data in this paper are from the UPI of the 2018 personality test of D University.

### 4.3. Applied Research

1. *Input*: the order of input samples is defined as sex, age, and 10 factors of the self-evaluation table

Table 2 lists the mental health data table of some college students in the database, as well as the corresponding values of 10 factors.

(2) *Data standardization processing*: standardizing the psychological test data of 2010 college students
(3) *Set the fuzzy factorMand the iteration termination conditionI*: according to a large number of experiments, set *M* = 3, *I* = 1*e* − 4
(4) *Determine the range of the initial cluster center*: determine the range of the initial cluster center value [Cmin, Cmax]. In general, Cmin = 3, Cmax = √*n*; there are 2010 groups of data in this experiment. The minimum value of the number of fuzzy clustering Cmin is 3, and the maximum value of fuzzy clustering number *C* is 10
(5) *Define the initial cluster center*: in the process of increasing the number of cluster centers from Cmin to Cmax, calculate the cluster center corresponding to each cluster number *C*
(6) The deviation degree of sample points is calculated and the transition value of information entropy is calculated
(7) Determine the weight and adjust the verification cluster center

## 5. Results and Discussion

### 5.1. FCM Algorithm and FCM Algorithm Based on Information Entropy Attribute Weighting

The FCM collection algorithm based on information entropy customization is used to analyze the mental health data of college students. The assembly results are compared with the traditional FCM clustering algorithm, and its effectiveness is confirmed by tests. According to the determination of the final clustering company and the impact of the 10 factors on the cluster results, the models are divided into four categories.

As shown in Figure 1, the projectiles generated by the FCM algorithm and the FCM algorithm based on the density of information entropy characteristics are compared. The more repetitions, the lower the collection efficiency. In contrast, the more repetitive, the greater the efficiency of compilation. The number of iterations of the FCM algorithm based on the density of information entropy characteristics is less than that of the FCM algorithm, which indicates that the performance of the FCM algorithm is improved and the overall performance of the FCM algorithm is better than that.

### 5.2. Cluster Results of College Students' Mental Health

As shown in Figure 2, the results of the mental health consolidation of college students in 2010 are as follows: 104 students are in the first category, representing 5.2% of the total. There are 474 students in the second category, representing 23.6% of the total. 728 students are in the third category, representing 36.2% of the total. There are 749 students in the fourth grade, representing 37.3% of the total.

### 5.3. Mental Health Status of Four Types of Students

As shown in Figure 3, the mental health status of the freshmen of grade 2018 and 2010 in D University is as follows: 151 (6.45%) have poor psychological quality, 463 (22.28%) have poor psychological quality, and 1468 (71.67%) have good psychological quality. There are 614 students with psychological problems, accounting for 28.73% of the total.

### 5.4. Analysis of Mental Health Data

As shown in Figure 4, the FCM algorithm based on information entropy customization is used to analyze students' mental health data to determine whether there are significant differences between the various factors and then the extent of each effect factor on a set of results.. You can see from Figure 4 that anxiety, sensitivity, and psychosis have the highest effect on cognitive effects, while somatization and other factors have the least effect on cognitive effects. We suggest that the school mental health counseling center pay special attention to the prevention and direction of stress and self-attraction of participants, according to the classification of mental health conditions, based on the characteristics of different psychological problems, for different treatment, targeted psychological intervention, or health education.

## 6. Conclusion

This article applies the method of cluster analysis to the mining and research of the main factors of college students' mental health, which is a beneficial discussion. Student mental health education is a new complex program and project. Only by reforming the students' mental health education system, transforming the mental health education of students and improving the teaching methods and ability to guide staff, can we contribute to their development. Staff must switch from nonprofessional to professional, and content and approach must change to make mental health services easier to explore and develop basic skills. College educators should analyze the current situation and existing mental health problems of college students from sound perspectives, using both scientific knowledge to understand the developmental culture of disciplining mental health education and guidance in stimulating mental health quality as the underlying cause. Finally, college educators must not only rely on mental health care but also pay attention to prevention and deep concern for the inner life of college students. In order to adapt to the rapid development of society, students focus on the speed and speed of learning, and life and their spiritual pressures increase, which will lead to negative learning. With the continuous development of education in China, a variety of research in favor of the development of education is emerging nonstop, which greatly promotes the sustainable development of education. For any type of mental health problem, educational measures must be taken that should analyze the reasons in anticipation, in order to manage the psychological problems that students have, so that students will have good physical and mental conditions to conform to college life and to have the right views of life, values, and worldview.

The clustering analysis algorithm is applied to the analysis of college students' mental health. Through the clustering analysis algorithm, the common rules and problems existing in the mental health of college students are found, so as to correctly manage and educate students. The main results of this paper are as follows: the cluster analysis algorithm is applied to the analysis of college students' mental health, which is an effective analysis of mental health data. The FCM algorithm and the FCM algorithm based on information entropy attribute weighting are used to study the influence of mental health factors on the clustering results, and the practicability of the algorithm is obtained, which provides a reference for college students to prevent mental health problems in the early stage. In the two-step clustering analysis algorithm, it is necessary to further study the influence of parameter settings on the algorithm. Master the characteristics and rules of parameter setting, so that the algorithm can get the best performance. For the collection of college students' mental health data, professional knowledge should be further used to explore the influencing factors on mental health, so as to make the prediction more accurate. In a word, it does have a certain role in diagnosing and finding the cause of mental health diagnosis, but it also has certain limitations. As long as we can recognize these limitations and pay attention to avoid the diagnostic deviations caused by their limitations in actual use, this will surely provide us with valuable information in mental health diagnosis and become effective in the mental health diagnosis of college students.

## Figures and Tables

**Figure 1:** Comparison of objective functions.

**Figure 2:** Cluster analysis of college students' mental health.

**Figure 3:** UPI tests the distribution of class personnel in each department.

**Figure 4:** Analysis of variance of mental health factors.

**Table 1:** Student's attribute code table.

Attribute	Gender	Family income	Single parent family	Only child's performance	Grade	Personality characteristics
Attribute value	Female	High	Yes	Yes	Excellent	Introverted rational type
Code	21	41	61	51	71	24

**Table 2:** Data table of mental health database for college students.

Gender	Age	Department	Somatization	Obsessive compulsive symptoms	Interpersonal sensitivity	Depressed	Anxious	Paranoia	Hostile	Psychotic	Other
Male	22	Foreign languages	1.17	1.9	1.77	1.53	1.2	1.67	1.54	1.3	1.34
Female	21	Chinese language	1.56	1.7	2	1.72		1.67	1.33	1.6	1.54
Male	21	Computer science	1.91	1.6	2	1.89	1.5	1.67	1.83	1.7	1.34
Female	20	Chemical engineering	2.25	2.4	2.21	1.62	2	1.67	1.34	1.5	1.7
Female	20	Economic management	1	1.1	2.11	1.23	1.8	1.17	1	1.4	1.29
Male	21	Civil engineering	1.08	1.7	1.9	2.07	1.9	1.5	1.67	1.8	1.4
Female	20	Social science	1.33	1.6	2.11	1.15	1.3	1.67	1.33	1.4	1

## Data Availability

The data that support the findings of this study are available from the corresponding author upon reasonable request.
